This article has been retracted.

# Modeling and Analysis of the Relationship between Aerobic Exercise and Obesity Reduction in Adolescents

**DOI:** 10.1155/2022/9957916

**Published:** 2022-03-21

**Authors:** Nan Fu, Kesen Li

**Affiliations:** ^1^Yunnan Technology and Business University, Yunnan, Kunming 650000, China; ^2^Dianchi College of Yunnan University, Yunnan, Kunming 650228, China

## Abstract

In order to solve the relationship between youth aerobic exercise and obesity reduction, an improved ant colony algorithm-oriented aerobic exercise method was proposed. Firstly, the changes in body shape, weight, BMI, body fat, body circumference, and other indicators of obese adolescents before and after aerobic exercise were used as the initial pheromone distribution matrix, and the random evolution factor and evolutionary drift threshold were introduced to establish the target function of reducing obesity caused by aerobic exercise in adolescents. The constraint conditions of the relationship between aerobic exercise and adolescent obesity reduction were explained, and the particle algorithm was introduced to establish the optimal model of aerobic exercise for adolescent obesity reduction. The experimental results show that with the increasing number of experiments, the advantages of this method are more obvious. From the overall level, the average modeling error of this method is about 0.053%, while the average error of the traditional method is about 0.186%, which shows that this method can control the error within a reasonable range, and it is proved that the improved ant colony algorithm can have a good correlation with the method of aerobic exercise.

## 1. Introduction

Adolescence is the period before the development of secondary sexual characteristics. Puberty occurs between the ages of 11 and 16 for girls and 6 and 13 for boys. People are very concerned about the healthy growth of teenagers [1]. Therefore, in order to meet the growth and development needs of teenagers, it is necessary to provide children with a lot of nutrition and increase energy intake. In recent years, the trend of adolescent obesity has become more and more serious, which has attracted close attention from parents, schools, society, and relevant experts [2]. According to an expert survey, the proportion of overweight and obese urban students is 12.03 percent, and it is increasing by 8 percent every year. More and more children and adolescents' health is damaged by obesity. Many children with overweight problems have one or more risk factors for cardiovascular diseases, so parents and teachers should actively help their children participate in weight loss activities. Obese adolescents eat too much fat, protein, and carbohydrates and they are reluctant to eat vegetables, and their nutrient intake is very uneven. Many eat more and exercise less which causes weight gain which further leads to all kinds of chronic diseases and endanger the health of children. The negative effects of childhood and adolescent obesity and inactivity on children's health include high blood pressure, atherosclerosis in adolescents, and type 2 diabetes in adolescents.

Among obese adolescents, the most common health-related goal is to lose weight, and a well-designed aerobic endurance exercise training program can help teens better achieve this goal. Aerobic exercise is considered one of the easiest and most effective ways to lose weight. It refers to a physical exercise which helps the body to get fully oxygenated and achieve a physiological balance. To put simply, aerobic exercise refers to any rhythmic exercise with a long duration of exercise (about 15 minutes or more) of light to moderate intensity (75 to 80 percent maximum heart rate). The most important aerobic training in sports are the common aerobic exercise forms, which are walking, jogging, swimming, running, aerobics, cycling, climbing, jumping rope, basketball, football, and so on. The purpose of aerobic exercise is to build up cardiorespiratory endurance. Li. J. conducted an experimental comparison of 100 students before and after learning aerobics for one year and performed a rational analysis of the questionnaire survey results. Before aerobics training, the 100 students were with slightly obese figure with an average body fat of 32.1%; after a year of aerobics training, they reached the standard level. Their body fat volume fell by 6% and on average was 26.1%. Before exercise, 50 or so students were beyond the normal standard and they exercised light for fueling posture, 90% of them were standard type after exercise, and the average body fat volume decreased from 15 kg before exercise to 12.5 kg after exercise, and the average fat volume of each person decreased by 2.5 kg [3]. Berge. J. divided 60 girls into two groups according to age and height. The exercise time of the high-intensity exercise group was 40–60 min, including 5 min of preheating, 10 min of forming posture exercise, and 20–30 minutes of running or pedal exercise. The low-intensity exercise group was 40–60 min, including 5 min of dynamic warming up, 15 min of exercise, and 15–20 min of calisthenics. Studies have shown that calisthenics can effectively reduce weight and improve body shape when the exercise is more powerful. When the exercise time and intensity of calisthenics increase, it can also improve the utilization rate of fat, reduce body fat, and increase muscle strength [4]. A. Garcia-Hermoso conducted a questionnaire survey of 981 middle school students from 10 middle schools. SPSS data analysis results showed that physical exercise factors had a direct and indirect relationship with the self-esteem of middle school students. Exercise intensity has a very important influence on the improvement of self-confidence in middle school students [5]. To solve the above problems, an improved ant colony algorithm was proposed to model the relationship between aerobic exercise and adolescent obesity reduction. Compared with traditional methods, this paper combines the improved ant colony algorithm with evolutionary factors and combines the evolutionary drift threshold to set up the relationship between obesity and aerobic exercise in adolescents. In order to reduce the constraint range of modeling, within the constraint range, the establishment of adolescent obesity aerobic exercise model is simplified by particle swarm optimization (PSO) algorithm, which avoids the shortcomings of traditional methods. Finally, its performance is verified by simulation [6].

## 2. Modeling Principle of the Relationship between Aerobic Exercise and Obesity Reduction in Adolescents

For modeling the relationship between aerobic exercise and adolescent obesity reduction process, the first step is acquisition of teenagers suffering from various factors of obesity. Then calculate the weights of various factors on the adolescent health damage coefficient and set up aerobics constraint model for the relationship between the adolescent obesity and aerobic exercise. Aerobic exercise is given on the relationship of the adolescent obesity to reduce constraints. Calculate the objective function; the function is used to solve the problem model and establish the model. The specific steps are described as follows.

Assuming that *Q*_*s*_ represents the main causes of obesity and *x*_*i*_*w*_*i*_ represent the psychological and physical harm caused by obesity to adolescents, the following formula is used to calculate the weight coefficient of the harm caused by each obesity hazard factor to the physical health of adolescents:

(1) $$\begin{array}{c} q_{h}=\frac{\left(Q_{s}\cdot \lambda \right)}{x_{i}\cdot w_{i}}\times \varepsilon \left(Q\cdot \beta \right). \end{array}$$

Here, *ε* represents the number of fat cells in the body, *Q* represents the increase period of fat content in the cells of obese youth, and *β* represents the calorie intake of obese youth [7].

The relationship constraint model of aerobic exercise on the reduction of adolescent obesity was established and expressed by the following formula:

(2) $$\begin{array}{c} Q_{rij}\left(t+n\right)=\frac{\left(1-\rho \right)\cdot Q_{rij}\left(t\right)}{q_{h}}. \end{array}$$

Here, *ρ* represents changes in body shape and body composition of obese adolescents before and after exercise, and *Q*_*rij*_(*t*) represents comprehensive risk factors for cardiovascular and other pathological changes of obese adolescents [8].

Assuming that *τ*_*ij*_(*t*+1) represents the constraint conditions of the relationship between aerobic exercise and adolescent obesity reduction, and *TP* represents the state of adolescent obesity, the following equation is used to calculate the objective function of the relationship between aerobic exercise and adolescent obesity reduction:

(3) $$\begin{array}{c} Q^{*}=Q_{rij}\left(t+n\right)\times \frac{FN}{TP}\cdot FP\tau_{ij}\left(t+1\right). \end{array}$$

*FP* represents the change in blood pressure before and after exercise, and *FN* represents the decrease in waist and hip circumference of obese adolescents after exercise. However, the traditional methods cannot obtain the changes of various indicators of obese adolescents before aerobic exercise, which reduces the accuracy of the model. An improved ant colony algorithm was proposed to model the relationship between aerobic exercise and adolescent obesity reduction [9].

## 3. Modeling of the Relationship between Aerobic Exercise and Obesity Reduction in Adolescents

### 3.1. Objective Function: Acquisition of the Relationship between Aerobic Exercise and Obesity Reduction in Adolescents

In the optimization modeling process of adolescent obesity aerobic exercise reduction, firstly, the ant colony algorithm is used to converge the changes of body shape, weight, BMI, body fat, body circumference, and other indicators of obese adolescents before and after aerobic exercise as the initial pheromone distribution matrix, and then the random drift progression factor and evolution threshold are introduced to establish the objective function. It also explains the constraint conditions that aerobic exercise needs to be satisfied in reducing the relationship between obesity in adolescents, and the specific steps are described as follows.

It is assumed that *q*_*ij*_ represents the change factors of body shape information of obese adolescents before and after aerobic exercise. A represents the influence of obesity on the activity level of adolescents, and ∂_*ij*_ represents the change factors of BMI index of obese adolescents before and after aerobic exercise. The following formula is used to establish the initial distribution matrix of pheromone represented by *η*_*ij*_ integrating the following ant colony algorithm:

(4) $$\begin{array}{c} \eta_{ij}=\frac{\left(q_{ij},M_{ij}\right)\times A}{\left(\partial_{ij},d_{ij}\right)\times R_{ij}}\times K_{ij}. \end{array}$$

Among them, *M*_*ij*_ represents the energy accumulation state of obese adolescents before and after exercise, and *d*_*ij*_ represents the change factors of low-density lipoprotein secretion information of obese adolescents before and after exercise. According to the principle of the ant colony algorithm, random evolutionary factors and evolutionary drift threshold were introduced to calculate the objective function of the relationship between aerobic exercise and adolescent obesity reduction in the process of establishing the optimization model of the relationship between aerobic exercise and adolescent obesity reduction, and its constraint conditions were given [10]. The evolutionary drift threshold is defined as the variation threshold of the probability of ants selecting the next path node, and the random evolution factor is defined as the probability variation parameter of ants selecting the next path node. The specific steps are detailed as follows:

(1) It is assumed that each ant represented by REF_*k*_ will be assigned a probability value. When the REF_*k*_ value is higher than the weight coefficient of the influence of obesity on adolescents represented by EDT, the following equation is used to establish the probability model of reducing obesity of adolescents by aerobic exercise:

(5) $$\begin{array}{c} p_{ij}^{k}\left(t\right)=\left\{\begin{array}{c} \frac{\tau_{ij}^{\alpha }\left(t\right)\cdot \eta_{ij}^{\beta }\left(t\right)}{\tau_{ij}^{\alpha }\left(t\right)\cdot \eta_{ij}^{\beta }\left(t\right)}\\ {\text{REF}}_{k}\geq \text{EDT} \end{array}\right), \end{array}$$

where *τ*_*ij*_(*t*) represents the coefficient of difference between the body shape of obese adolescents and that of adolescents with normal physical fitness, *α* represents the relative importance of residual information, *β* represents the relative importance of expected value, and *η*_*ij*_(*t*) represents the probability value obtained by each ant of reducing adolescent obesity by probability aerobic exercise [11].

(2) Among the optimal solutions found by each generation of ants, *R*_*ij*_ represents the subpath, and the following formula is used to search out the path whose contribution degree of *R*_*ij*_ to the overall optimal path is greater than the path contribution threshold:

(6) $$\begin{array}{c} {\text{CDSP}}_{ij}=\frac{R_{ij}\cdot D\left(i,j\right)}{L_{i}}p_{ij}^{k}\left(t\right), \end{array}$$

where *D*(*i*, *j*) represents the optimal solution neutron path, and *L*_*i*_ represents the ant colony finding the optimal solution of this iteration after the *i* iteration.

The following equation is used to establish the objective function of the relationship between aerobic exercise and adolescent obesity reduction:

(7) $$\begin{array}{c} \Delta \tau_{ij}\left(\text{enforce}\right)=\frac{\Delta \tau_{ij}\left(\text{new}\right)+\Delta \tau_{ij}}{{\text{CDSP}}_{ij}\cdot q_{0}}\times p_{ij}^{k}\left(t\right), \end{array}$$

where Δ*τ*_*ij*_ represents the first update of pheromone on the optimal solution neutron path (*i*, *j*), *q*_0_ represents the path contribution threshold, and Δ*τ*_*ij*_(new) represents the final total pheromone amount on the path (*i*, *j*) [12].

The following formula is used to provide the constraint conditions that aerobic exercise needs to meet to reduce adolescent obesity to constrain the objective function:

(8) $$\begin{array}{c} \Delta \tau_{ij}^{k}=\frac{{\text{CDSP}}_{ij}\times p_{ij}^{k}\left(t\right)}{\Delta \tau_{ij}\left(\text{enforce}\right)}\cdot \eta_{ij}\left(t\right). \end{array}$$

In conclusion, in the process of optimal modeling of reducing obesity caused by aerobic exercise, the ant colony algorithm integrated with the ant colony algorithm first used the changes in body shape, weight, BMI, body fat, body circumference, and other indicators of obese adolescents before and after aerobic exercise as the initial pheromone distribution matrix. Random evolutionary factors and evolutionary drift threshold were introduced to establish the objective function of reducing adolescent obesity by aerobic exercise, and the constraint conditions for reducing adolescent obesity by aerobic exercise were explained, which provided the basis for establishing the model.

### 3.2. Modeling the Relationship between Aerobic Exercise and Obesity Reduction in Adolescents Based on Particle Algorithm

In the process of optimal modeling of the relationship between aerobic exercise and adolescent obesity reduction, the particle algorithm is introduced to establish the optimal model based on the objective function of the constraint conditions that aerobic exercise needs to meet for adolescent obesity reduction given in the above formula. The specific steps are described as follows.

Suppose that *X*_*i*_=(*x*_*i*1_, *x*_*i*2_,…, *x*_*i*  *D*_) is based on *i* obtained by the above formula representing the Δ*τ*_*ij*_^*k*^ particle, and the best position (with the best fitness value) it has experienced is expressed as follows:

(9) $$\begin{array}{c} p_{i}=\frac{\left(P_{i1},P_{i2},\ldots ,P_{i\;D}\right)}{X_{i}=\left(x_{i1},x_{i2},\ldots ,x_{i\;D}\right)}\times \Delta \tau_{ij}^{k}, \end{array}$$

where *P*_*i*1_, *P*_*i*2_, and *P*_*i*  *D*_, respectively, represent the historical optimal position through which the particle passes.

Assuming that GBEST represents the index number of the best position through which all the particles in the swarm pass, the velocity of the particles is expressed by the following formula:

(10) $$\begin{array}{c} V_{i}=\frac{g\text{best}\cdot P_{i}}{\left(v_{i1},v_{i2},\ldots ,v_{i\;D}\right)}. \end{array}$$

For *d* dimension of each generation of particles, the following formula is used:

(11) $$\begin{array}{c} v_{i\;d}\left(t+1\right)=v_{i\;d}\left(t\right)+c_{1}r_{1}\left[p_{i\;d}-x_{i\;d}\left(t\right)\right]+c_{2}r_{2}\left[p_{p\;d}-x_{i\;d}\left(t\right)\right], \end{array}$$

where *c*_1_ and *c*_2_ stand for normal numbers, which are two random numbers varying within [0,1] range, *t* and *t*+1 stand for algebra, *v*_*i*  *d*_ stands for the speed of each particle in *d* dimension, I stands for particle number, *d* stands for dimension, and *r*_1_*r*_2_ stand for a random number between 0 and 1. *p*_*i*  *d*_ represents the best position that each particle has been in so far, *p*_*g*  *d*_ represents the optimal position of all particles so far, and *x*_*i*  *d*_ represents the current position of the particle.

The following equation is used to establish the relationship between aerobic exercise and obesity reduction in adolescents:

(12) $$\begin{array}{c} \min f\left(x\right)=\frac{v_{i\;d}\left(t+1\right)\times V_{i}}{X_{i}}. \end{array}$$

## 4. Simulation Results and Analysis

The subjects of the experiment were recruited from the young people who voluntarily participated in aerobic exercise to lose weight. With an average age of 14–19 years old, a total of 60 obese adolescents, including 30 males and 30 females, underwent low-intensity long-term aerobic exercise for 6 weeks. Informed consent was required to be signed by the parents of the subjects before the experiment. The test indexes mainly include four blood lipids: high-density lipoprotein cholesterol (HDL-C), low-density lipoprotein cholesterol (LDL-C), total cholesterol (TC), and triglyceride (TG), which are tested by enzyme method. Blood glucose indicators fasting blood glucose (FPG), blood glucose two hours after meal (2hPG), and glycosylated hemoglobin (HbAIC) were tested by glucose oxidase method.

### 4.1. Accuracy Comparison of Different Modeling Methods

The improved algorithm, neural network, and fuzzy theory were used to model the relationship between aerobic exercise and adolescent obesity reduction, and the modeling experiment of aerobic exercise on adolescent obesity reduction was conducted to observe the changes in body shape and body composition of adolescents before and after aerobic exercise. The statistical results of the two different algorithms were compared with the average changes in the body shape and body composition of the adolescents before and after aerobic exercise, and the comprehensive effectiveness of the two different models was evaluated by the comparison results. The comparison results are shown in Tables 1 and 2.

By analyzing Tables 1 and 2, it can be seen that when the method in this paper is used to analyze the changes in index values of obese adolescents before and after aerobic exercise, the changes in index values obtained by this method are basically consistent with the actual values, while the gap between the traditional method and the actual values is large, indicating that the modeling method in this paper has high accuracy.

### 4.2. Error Comparison of Different Modeling Methods

The relationship between aerobic exercise and adolescent obesity reduction was modeled by improved algorithms, neural networks, and fuzzy theory, respectively. Under different experiments, the error rate of two different algorithms to establish the model of aerobic exercise to reduce adolescent obesity was compared.  Figure 1 shows that under the same experimental conditions, the method of modeling error is far less than the neural network and fuzzy theory of aerobic exercise on the relationship of adolescent obesity to reduce modeling method of the traditional method; with the increasing the number of experiments, the advantages of this method are more obvious. From the overall level, the average modeling error of this method is about 0.053%, while the average value of the traditional method is about 0.186%, indicating that the error can be controlled within a reasonable range.

### 4.3. Influence of Long-term Aerobic Exercise on Lipids of Obese Adolescents

Figures 2–5, respectively, describe the changes of TC, LDL-C, TG, and HDL-C in male and female subjects before and after long-term aerobic exercise.

It can be seen from Figures 2–5 that after 6 weeks of aerobic exercise, the TG and LDL-C values of male subjects were significantly lower than those before exercise, *P* < 0.01; TC value was significantly lower than before exercise, *P* < 0.05. There was no significant difference in HDL-C (*P* > 0.05). The TG, TC, and LDL-C values of female subjects were significantly lower than those before aerobic exercise, but there was no significant difference in HDL-C values.

## 5. Conclusion

An improved ant colony algorithm-oriented aerobic exercise method was proposed. In the analysis of index changes of obese adolescents before and after aerobic exercise, the obtained index changes were basically consistent with the actual value, while there was a large gap between the traditional method and the actual value. The average error of the proposed method is about 0.053%, while that of the traditional method is about 0.186%. It shows that the proposed method can control the error within a reasonable range, and the improved ant colony algorithm aerobic exercise method can well explain the relationship between the two.

## Figures and Tables

**Figure 1:** Comparison of modeling errors of different algorithms.

**Figure 2:** TG changes in male and female subjects before and after aerobic exercise.

**Figure 3:** Changes in TC of male and female subjects before and after aerobic exercise.

**Figure 4:** Changes in HDL-C in male and female subjects before and after aerobic exercise.

**Figure 5:** Changes in LDL-C in male and female subjects before and after aerobic exercise.

**Table 1:** Changes of index values before exercise by different methods.

Index	Improved method	Actual value	Traditional method
stature	170	170	170
weight	103.3	103.3	103.3
BMI	34.77	34.77	34.77
Waist	106.3	106.29	106.29
Hipline	118.9	118.89	118.89
body fat rate	32.59	32.589	32.589
fat mass	11.09	11.08	11.08

**Table 2:** Changes of index values after exercise by different methods.

Index	Improved method	Actual value	Traditional method
Stature	172.2	172.1	166.1
Weight	93.8	93.7	83.7
BMI	31.4	31.39	21.39
Waist	95.24	95.239	105.239
Hipline	102.5	102.4	112.4
body fat rate	34.12	34.11	34.11
fat mass	9.01	9.01	15.01

## Data Availability

The data used to support the findings of this study are available from the corresponding author upon request.
